RETRACTED

# Deep Learning-Based Three-Dimensional Oral Conical Beam Computed Tomography for Diagnosis

**DOI:** 10.1155/2021/4676316

**Published:** 2021-09-21

**Authors:** Yangdong Lin, Miao He

**Affiliations:** Tianjin First Central Hospital, Tianjin 300192, China

## Abstract

In order to deeply study oral three-dimensional cone beam computed tomography (CBCT), the diagnosis of oral and facial surgical diseases based on deep learning was studied. The utility model related to a deep learning-based classification algorithm for oral neck and facial surgery diseases (deep diagnosis of oral and maxillofacial diseases, referred to as DDOM) is brought out; in this method, the DDOM algorithm proposed for patient classification, lesion segmentation, and tooth segmentation, respectively, can effectively process the three-dimensional oral CBCT data of patients and carry out patient-level classification. The segmentation results show that the proposed segmentation method can effectively segment the independent teeth in CBCT images, and the vertical magnification error of tooth CBCT images is clear. The average magnification rate was 7.4%. By correcting the equation of *R* value and CBCT image vertical magnification rate, the magnification error of tooth image length could be reduced from 7.4. According to the CBCT image length of teeth, the distance *R* from tooth center to FOV center, and the vertical magnification of CBCT image, the data closer to the real tooth size can be obtained, in which the magnification error is reduced to 1.0%. Therefore, it is proved that the 3D oral cone beam electronic computer based on deep learning can effectively assist doctors in three aspects: patient diagnosis, lesion localization, and surgical planning.

## 1. Introduction

With the rapid development of information technology, a large amount of data has been accumulated in various fields. In the medical field, more and more data sets have been collected, especially medical image data sets [1]. In recent years, deep learning has made great breakthroughs in the field of natural image processing, which can achieve good results in many tasks. More and more researchers are applying deep learning technology to medical image processing. However, most of the current medical image studies are focused on two-dimensional images and most of the parts studied are concentrated on human viscera and eye areas [2]. Digital technologies such as CAD/CAM, rapid prototyping, and “3D printing” are all based on CT and CBCT image data for reference in the aspects of intelligent processing of dental prostheses and the production of accurate dental implant guide plates. In the aspect of modeling, the three-dimensional finite element model of the prosthesis and the soft and hard tissues of the tooth collar can make the analysis of oral biomechanics more intuitive with the help of CT anatomical data. In addition, in the aspect of measurement, CBCT three-dimensional image data are often used for accurate measurement of the cranial surface, including bone defect volume and tooth length measurement. Therefore, the image data derived from CT are the basis of intelligent oral prosthesis, accurate implantation, and finite element mechanical model; if the data are not accurate, the reliability of the calculation results, conclusions, and clinical efficacy will be greatly reduced [3]. Therefore, it is important to understand the differences between CBCT data and real data. In this study, we studied the deep learning-based diagnosis of neck and facial diseases in order to meet the challenges of 3D cone beam computed tomography (CBCT) data. In terms of patient classification, this paper proposes a deep diagnosis of oral and maxillofacial diseases (DDOM) [4] and tooth segmentation network (TSNet) [5] based on deep learning. Different from the current algorithm which can only classify two-dimensional images, the DDOM algorithm proposed in this paper can process the three-dimensional oral CBCT data of patients and conduct patient-level classification. The results on a real data set containing oral CBCT data from 2500 patients show that the present method is superior to that of most specialists. In the aspect of tooth segmentation, compared with existing tooth segmentation algorithms, the algorithm uses convolutional neural network and adversarial network. The results on a real data set containing 100 oral CBCT images show that the proposed method achieves better tooth segmentation accuracy than existing methods [6].

RETRACTED

Fan et al. proposed a deep CNN-based automatic tooth instance segmentation method, called ToothNet framework, whose network structure consists of two networks. The first network extracts the edge image from the input CBCT image, enhances the contrast of the shape boundary, and then transmits the edge image and the input image to the second network; in the second network, the ToothNet network is constructed based on the 3D region proposal network, and the new learning similarity matrix is adopted. In order to effectively remove redundancy, accelerate training, and save GPU memory, at the same time, the tooth spatial relationship is encoded as additional feature input in the recognition task to improve the recognition accuracy. The method can automatically generate accurate segmentation and recognition results of tooth examples and is superior to the most advanced methods. This method firstly uses CNN to segment and recognize teeth in CBCT images [7]. Kothari et al. evaluated the CNN algorithm in the detection and diagnosis of dental image diseases, and the results showed that the deep CNN algorithm achieved a very good performance in the detection and diagnosis of dental image caries diseases [8]. Li et al. proposed a new deep learning framework for automatic labeling of anatomical sites in CBCT images [9]. It is necessary to explore how to use artificial intelligence technology to build a powerful image intelligent diagnosis platform and how to solve the contradiction between the surge in the number of images and the shortage of doctors, so as to improve the efficiency of image diagnosis and reduce the phenomenon of missed diagnosis and misdiagnosis. The current research on the above problems is insufficient. On the basis of current research, we studied the deep learning-based diagnosis of neck and facial diseases to meet the challenges of 3D cone beam computed tomography (CBCT) data. As far as we know, this is the first time to study the diagnosis of diseases in oral neck and facial surgery based on deep learning [10].

## 2. Methods

### 2.1. Image Classification Task

The task of image classification is to classify unknown images so as to get their accurate marks. As the first image task is to use deep learning, there are a variety of neural networks for image classification. Among all kinds of neural networks, convolutional neural network is the most frequently used neural network in image classification task [11]. Inception was proposed by Google in 2014, and the GoogLeNet at its core was the winner of the 2014 ImageNet competition. Inception network is a complete series that includes Inception v1, Inception v2, Inception v3, Inception v4, and Inception ResNet. Here, we will introduce the original Inception v1.

Inception v1: the core idea is that convolution at each level considers the use of multiple size convolution kernels at the same time, rather than using a single size convolution kernel at each level as previously reported. This structure is also known as an Inception module, and Figure 1 shows an example of one. In fact, this idea is similar to the “Network in Network” proposed in 2014, which is to make the submodules of the network become a small network. In this way, each layer of the network can be widened, so as to improve the fitting ability of each layer of the model and the overall fitting ability of the network.

However, in the original Inception network structure, due to Inception modules, the number of channels of the resulting feature graph at each layer would grow rapidly, which would make the model very large and would incur significant computational and memory overhead. Thus, the Google researchers proposed a dimensional reduction version of the Inception module, as shown in Figure 2. The main change is to add a layer of 1 x 1 convolution layer, which is used to change the number of channels, so that the number of channels in the whole network will not grow rapidly and the complexity of the network will be controlled [12]. This structure is also widely used in later convolutional neural networks.

RETRACTED

### 2.2. 3D Medical Data

In 3D medical data, the lesion area usually occupies only a small part of the total 3D data, and it is difficult to obtain satisfactory experimental results by directly classifying the whole 3D data. Therefore, for 3D medical data, the current methods often need to extract the lesion area first and then carry out specific classification of the lesion area. A two-stage quasialgorithm was designed for the problem of brain microhemorrhage. Three-dimensional convolutional neural network is used in both the stages. The first stage is used to extract the lesion area, and the second stage is used to further classify the extracted area [13]. Compared with using only the lesion area, there are some other methods for classification combining the lesion area and the overall image. The multiscale convolutional neural network structure is used to classify the lesion area of pulmonary nodules so that the features extracted by classification not only contain the lesion information but also include the lesion information. It also contains a larger range of global information. Because of the large amount of information contained in the three-dimensional CBCT data of oral cavity, it usually takes a lot of time and energy for doctors to process. In the case of limited oral medical resources, every doctor often needs to deal with a large number of oral CBCT data, which is easy for doctors to make wrong judgments under tired state [14]. In view of the challenges posed to doctors by CBCT image data, a deep learning disease classification algorithm DDOM based on CBCT data of oral and facial surgery was proposed. The symbol definition, algorithm details, and experimental results will be introduced.

### 2.3. Training Steps

First, spatial factorization is used during the whole training process of the first stage; we will select all the patient image knives and divide them into two types: sick images and normal images to form the training data set of the first stage. When the image is fed into the above network, we will get a two-dimensional output. At this time, the two-dimensional output needs to be input into the normalized exponential function (Softmax) to get the probability of the current image corresponding to each class and then calculate the loss by combining the loss function. The loss function adopted by DDOM in the first stage of training is the cross-entropy loss function, and the specific calculation formula of the loss is shown as follows:

(1) $$\begin{array}{c} L\left({\hat{Y}}_{i},y_{i}\right)=-\log\left(\frac{\exp\left({\hat{Y}}_{i}\left[y_{i}\right]\right)}{\sum_{j=1}^{C}\exp\left({\hat{Y}}_{i}\left[j\right]\right)}\right)=-{\hat{Y}}_{i}\left[y_{i}\right]+\log\left(\overset{C}{\underset{j=1}{\sum }}\exp\left({\hat{Y}}_{i}\left[j\right]\right)\right), \end{array}$$

where *y*_*i*_ represents the actual marking category of the current sample *X*_*i*_, *y*_*i*_=1 represents the current sample *X*_*i*_, and it belongs to class *j*; ${\hat{Y}}_{i}$ represents the output obtained after the current sample *X*_*i*_ is input to the network, and it is a two-dimensional vector; ${\hat{Y}}_{i}\left[j\right]$ represents the output of the current sample *X*_*i*_ corresponding to class *j*; and *C* represents the total number of categories [15, 16]. Since the first stage is divided into diseased images and normal images, *C* = 2.

RETRACTED

The following gradient return formula (2) can be obtained according to the cross lineal loss function in the first stage:

(2) $$\begin{array}{c} \frac{\partial L\left({\hat{Y}}_{i},y_{i}\right)}{\partial {\hat{Y}}_{i}\left[j\right]}=\frac{\partial \left(-{\hat{Y}}_{i}\left[y_{i}\right]+\log\left(\sum_{j^{\prime }=1}^{C}\exp\left(\hat{Y}{\left[j^{\prime }\right]}_{i}\right)\right)\right.}{\partial {\hat{Y}}_{i}\left[j\right]}. \end{array}$$

Among them, ∏(*j*=*y*_*i*_) is an indicator function (Indicator Function), and specific expressions are as follows:

(3) $$\begin{array}{c} \prod \left(j=y_{i}\right)=\left\{\begin{array}{cc} 0 & j\neq y_{i}\\ 1 & j\neq y_{i} \end{array}\right\}. \end{array}$$

Because of the single image input, only the prediction results of the single image can be obtained according to the model of the first stage, but the prediction results of the whole patient cannot be obtained. So, we can get a prediction of all the images for each patient, and then we can sort all the images from head to head, find the maximum number of consecutive images per patient that can be identified as diseased [17, 18]. Then, a closed value was set, and the patients whose maximum continuous sheet number reached the threshold value were judged as sick patients; otherwise, they were judged as normal people.

Finally, we first use the ImageNet pretraining model to initialize the parameters of the model. Then, according to the cross-entropy loss function, the network parameters were constantly updated through BP algorithm, and the model with the highest patient accuracy was selected as the final classification model in the first stage [19]. The algorithm in the first stage mainly converts the 3D data into a number of continuous images, thus transforming the 3D problem into a 2D problem. Then, through the prior knowledge, the results of two-dimensional images are used to get the results of three-dimensional data (Algorithm 1).

RETRACTED

## 3. Experimental Analysis

Since our goal is to segment tumor images from oral CBCT data, the experimental part of this chapter still adopts oral CBCT data set. The data sets in this chapter are all directly obtained using two-dimensional CBCT images. Since the labeling cost of lesion segmentation is relatively high, 680 patients were selected for labeling. For each patient, we developed an image line label from each of his lesions. In the actual training, we divided the data set into training set, verification set, and test set in an 8 : 1 : 1 random division according to patients. Unlabeled data are only used in the training process, not in the testing process.

### 3.1. ASNet Algorithm

To evaluate the different methods, the average crossover ratio is used here in this chapter (mean Intersection over Union, referred to as “mIoU) as a final evaluation indicator. The calculation method of average crossover ratio can be expressed as follows:

(4) $$\begin{array}{c} mIoU=\frac{\left|P\cap Q\right|}{\left|P\cap Q\right|}. \end{array}$$

Among them, *P*={(*i*, *j*)} represents the set of points satisfying *Y*_*i*,*j*_=1 in the image. In the same way, *Q*={(*i*, *j*)} represents the set of points satisfying all ${\hat{Y}}_{i,j}>0.5$ in the mask.

The hardware environment used for the whole experiment is equipped with two Intel (R) Xeon (R) ES-2620 v4 CPU and 4 Titan XP GPU servers. At the same time, the PyTorch platform is used here to implement the antagonistic collaborative network.

During the training phase, we adjusted the size of all the images to 224 × 224 and flipped them randomly horizontally with a 50% probability. At the same time, we performed a random rotation of the image in the range of 10 degrees. In the test phase, we used the average of the predicted results of the two segmentation branches as the final segmentation results and used the ADAM gradient descent method to train the antagonistic cooperative network from random initialization. For the segmented network, we set the initial learning rate as LE-4. For the discriminant network, we set the initial learning rate as LE-SO. Meanwhile, we also set the weight attenuation coefficient of SE-5. In the training process, we trained a total of 150 rounds, and every 30 rounds attenuated the learning rate according to the following formula:

(5) $$\begin{array}{c} \text{learning rate}=\text{initial learning rate}\times {\left(1-\frac{\text{initial learning rate}}{\text{maximum number of rounds}}\right)}^{\beta }. \end{array}$$

Among them, *β* was set to 0.9 in the experiment. *λ*_`1_, *λ*_`2_,  and*γ* in the loss function are set to 0.01, 0.1, and 0.70, respectively.

RETRACTED

In the experiment, we also compare some of the most advanced semisupervised segmentation algorithms. Specifically, we choose semisupervised full convolutional neural network (SEMIFCN), spatial factorization, and ASNet (Algorithm 2) for comparison. These three methods are the most advanced semisupervised segmentation algorithms in medical images at present. At the same time, in order to verify the function of unlabeled data and antiloss function, we also carried out model simplification experiment in the experiment, where supervised ASNet without adv means that the antagonistic collaborative network only uses labeled data and does not use the antagonistic loss function. Supervised ASNet with adv represents that the adversarial collaborative network uses only tagged data and uses the adversarial loss function. ASNet without adv represents that the adversarial collaborative network uses all data, but does not use the adversarial loss function.

Figure 3 shows the test results from different methods trained with different amounts of labeled data. By comparing the adversarial collaborative network with semisupervised full convolutional neural network, spatial decomposition method, and ASNET, we can find that the adversarial collaborative network exceeds all other semisupervised segmentation networks and achieves the best effect on oral data set.

Table 1 shows the results of the model simplification experiment. By comparing the adversarial collaborative network with its variants, Supervised ASNet without adv, and supervised ASNet with adv, we can see that using unlabeled data does improve accuracy. By comparing the adversarial collaborative network with another variant and ASNet without adv, we can see that the adversarial loss function also contributes to improved accuracy.

Table 2 shows the test results obtained by training different methods with different amounts of labeled data. By comparing the adversarial collaborative network with semisupervised full convolutional neural network, spatial decomposition method, and ASNet, we can find that the adversarial collaborative network exceeds all other semisupervised segmentation networks and achieves the best effect on oral data set.

Table 3 shows the results of the model simplification experiment. By comparing the adversarial collaborative network with its variants, we can see that using untagged data does improve accuracy. By comparing the adversarial collaborative network with another variant, we can find that the counter loss function also helps to improve the accuracy.

RETRACTED

### 3.2. Result

In this study, we propose a new semisupervised medical image segmentation algorithm called adversarial collaborative network (ASNet). Adversarial collaborative networks can be trained with limited tagged data and large amounts of untagged data. Therefore, adversarial collaborative network can be effectively applied to medical image analysis where collecting large-scale labeled data is extremely difficult. The experiment on the segmentation task of oral tumor lesions shows that the antisynergistic network sting can achieve a better effect than other benchmark force methods. These benchmark methods include supervised learning and semisupervised learning.

## 4. Conclusions

The deep learning-based diagnosis of oral and facial surgical diseases is systematically studied. An algorithm is proposed for patient classification, lesion segmentation, and tooth segmentation, respectively. For patient classification, the proposed DDOM algorithm can effectively process the three-dimensional oral CBCT data of patients, and the segmentation results show that the proposed segmentation method can effectively segment the independent teeth in CBCT images, the vertical magnification error of tooth CBCT image was determined, and the average magnification rate was 7.4%. By correcting the equation of *R* value and CBCT image vertical magnification rate, the magnification error of tooth image length could be reduced from 7.4%. According to the CBCT image length of teeth, the distance *R* from tooth center to FOV center, and the vertical magnification of CBCT image, the data closer to the real tooth size can be obtained, in which average magnification rate is reduced to 1.0%. Therefore, this method can better assist doctors from three aspects of patient diagnosis, lesion location, and surgical planning.

The main problems and directions for further research are as follows: (1) restriction of data volume on research. Future studies need to expand the data set for further verification. Existing studies generally obtain the medical data related to oral cancer from cooperative hospitals with complicated procedures and great limitations. Although there is an oral cancer database in China, which has provided great help for the research of oral cancer, the database mainly focuses on biochemical information data, and there are few oral cancer image data. It needs to be replenished in the future. (2) Optimization of the model: the section map of oral cancer has its own characteristics. In the future, the differences and advantages of different algorithms can be explored, and different algorithms can be combined effectively to find the most suitable model for the identification of oral cancer. (3) Treatment of micrograph of oral carcinoma section: the processing method of oral cancer section map has greatly influenced the identification of oral cancer features by artificial intelligence. How to strengthen the oral cancer features in the picture and improve the efficiency of deep learning are also worthy of research.

RETRACTED

## Figures and Tables

**Figure 1:** Inception module.

**Figure 2:** Dimension reduction of the inception module.

**Figure 3:** Results of different methods using different amounts of labeled data on the test set.

**Algorithm 1:** First stage algorithm of patient classification.

**Algorithm 2:** ASNet algorithm.

**Table 1:** Results of model simplification experiment.

Method	10%	30%	50%	100%
Number of labeled data				
Supervised ASNet without adv	0.689	0.821	0.847	0.863
Supervised ASNet with adv	0.685	0.823	0.889	0.879
ASNet without adv	0.812	0.856	0.871	0.892
ASNet	0.832	0.865	0.871	0.906

**Table 2:** Results of different methods using different amounts of labeled data on the test set.

Method	10%	30%	50%	100%
Number of labeled data				
Supervised ASNet without adv	0.702	0.799	0.823	0.863
Supervised ASNet with adv	0.735	0.845	0.861	0.875
ASNet without adv	0.819	0.854	0.871	0.871
ASNet	0.837	0.865	0.872	0.906

**Table 3:** Results of model simplification experiment.

Method	10%	30%	50%	100%
Number of labeled data				
Supervised ASNet without adv	0.692	0.812	0.847	0.889
Supervised ASNet with adv	0.695	0.823	0.863	0.889
ASNet without adv	0.827	0.863	0.872	0.893
ASNet	0.837	0.865	0.872	0.906

## Data Availability

The data used to support the findings of this study are available from the corresponding author upon request.
